The article "Mechanical Analysis and Clinical Application of Butterfly-Shaped Patellar Claw" was retracted in 2023. Reasons: signs of a paper mill; compromised peer review; unreliable results or conclusions.

# Mechanical Analysis and Clinical Application of Butterfly-Shaped Patellar Claw

**DOI:** 10.1155/2022/2008668

**Published:** 2022-02-03

**Authors:** Yi Liu

**Affiliations:** Department of Orthopedics, The First People's Hospital of Fuyang Hangzhou, Hangzhou 311400, China

## Abstract

Memory alloy patella claws for treating patella fractures have been used for more than 30 years with many desirable features including fast healing, quick recovery, and avoidance of top abrasion of Kirschner wires and other complications. However, there are many models and it is difficult to choose the accurate claw for the patient. In this study, a finite element model of the butterfly-shaped patellar claw made of shape memory alloy was established, its mechanical structure was analyzed, and its clinical application was monitored. We used Solidworks Simulation software for modeling and mainly analyzed the force of the compression ring of the butterfly-shaped patellar claw. Clinically, we chose a closed fresh patella fracture case. After finite element analysis, the maximum stress that the compression ring of the butterfly-shaped patellar claw can withstand is 568.1 MPa. In this range, it always has elastic deformation resistance. The butterfly-shaped patella claw is fixed on the patella and will not break when subjected to a maximum force of 150 N on the encircling arm, and at the same time, there will be no pressure failure due to plastic deformation. A total of 27 cases were clinically used for the assessment of the clinical efficacy of the newly designed butterfly-shaped patella claws. The average follow-up time was 15.5 months, and the average fracture healing time was 8-12 weeks. All patients can get out of bed with crutches within 2 to 3 days after surgery. Among them, there were 15 cases with excellent functional ratings, 10 cases with good ratings, 2 cases with acceptable ratings, and no cases with poor ratings. The designed butterfly-shaped patella claws can provide an effective method for the treatment of patella fractures.

## 1. Introduction

Patella fractures are intra-articular fractures of the knee where most of the cases represent separated and displaced following fractures. The incidence of patella fractures accounts for 1% to 2% of human fractures [1, 2]. At present, there are many internal fixation methods for the treatment of patella fractures. Among them, the common methods include Kirschner wire tension bands, screws, steel wire cerclage, titanium cable cerclage, memory alloy patella claw (patella concentrator), and silk purse-string suture [3, 4]. Memory alloy patella claws have been used to treat patella fractures for more than 30 years [5]. It conforms to the principle of tension band fixation, and the fixation is firm. In addition, it can allow patients to perform early functional exercises, the patients recover quickly after the operation, and there is no phenomenon such as the top abrasion of Kirschner wires after the operation [4, 6]. However, it still has shortcomings, and there are many models and it is difficult to choose accurately. In the process of fracture fixation and compression, only the grip of the upper and lower claw branches is available, and the longitudinal pressure is lacking [6]. In clinical settings, sometimes the fracture line is wider, or the dorsal patella opens [7]. In addition, it can cause postoperative internal fixation loosening, patellar claw slippage, uncoupling, fracture displacement, and local uplift deformity [8, 9]. Therefore, only the gripping force of the patellar claws is not strong enough to fix, and longitudinal pressure is also required. Titanium-nickel shape memory alloy (TiNi SMA) represents a class of “smart materials” characterized by superelasticity, shape memory effect, corrosion resistance, excellent fatigue behavior, acceptable biocompatibility, and high damping capacity. All these characteristics render the TiNi SMAs a promising material for clinical applications especially in orthopedics [10, 11]. In this study, we used the characteristics of TiNi shape memory alloy to design the body of the patellar claw as a hollow-shaped longitudinal compression device to solve these problems. We applied relevant software to analyze the finite element mechanical properties of the patellar claw, and the effect was satisfactory after the initial clinical application. We call the newly designed patella claw a memory alloy butterfly-shaped patellar claw (Chinese utility model patent number: ZL 2007 2 0005050.4, hereinafter referred to as butterfly-shaped patellar claw). The designed memory alloy butterfly-shaped patellar claw was in 27 cases for assessment of clinical efficacy.

## 2. Materials and Methods

Keeping in mind the advantages of high strength and memory properties of TiNi shape memory alloy, we designed the waist of the patellar claw into a hollow dumbbell-shaped compression ring. The butterfly-shaped patellar claw was designed as shown in Figure 1. The main size is set according to the size of the anatomical structure. Solidworks Simulation software was used for mechanical structure analysis. The butterfly-shaped patellar claws used in this study were all produced by Lanzhou Ximai Memory Alloy Co., Ltd.

### 2.1. Model Establishment

Due to the possibility of excessive displacement during analysis, the solver may produce a nonlinear solution, which is nonconvergent in the simulation software, and finally causes the solver to fail. Therefore, we set the patellar claw to fit the patella perfectly. Although this kind of thing does not happen in reality, this assumption does not prevent the force of the patella acting on the compression ring from being changed by the flexion and extension of the knee joint in the real situation.

The fully annealed fracture strength of the memory alloy was 895 MPa. When the patella claw is installed in the human body, the separation tension of the patella due to the flexion and extension of the knee joint is far less than the tensile strength of the material itself. Based on this, whether the compression ring in the patellar claw has sufficient yield strength has become the main focus of research for this test. Therefore, we did not establish a patella model, but only a patella claw model. Through the above analysis of the model, we made the following settings:

1. The encircling claws of the patella claw could tightly fasten the outer edge of the patella
2. We did not consider the sliding between the patellar claw and the patella along the axis of the patella due to failure
3. We only analyzed the deformation of the compression ring, so the patella claw model was simplified and the encircling claw was hidden, as shown in Figure 2
4. The material of the patellar claw was TiNi memory alloy, as shown in Figure 3
5. To ensure that there is no penetration error in each structure during the solution process, the contact mode of the parts in the connection was set as joint
6. We constrained the degrees of freedom of the two lower jaws and load a roller/slider to fix the pressure ring to prevent the model from rotating in the radial direction during the simulation, as shown in Figure 4

### 2.2. Loading and Grid Control

Since the flexion and extension of the human knee joint will produce a maximum force of about 150 N on the patella (as shown in Table 1 [1]), a force of 150 N tangential to the patella claw was applied to the three claws of the patella claw, as shown in Figure 5.

In our simulation, we focused on analyzing the stress, strain, and displacement acting on the compression ring when the patella is separated. At the same time, to speed up the analysis time of the solver, the model meshed, and the length of one side of the square was kept 0.4 mm, as shown in Figure 6.

Considering that the shape of the compression ring at the joint of the beam changes greatly, the analysis result may not converge or the analysis result may be shifted in this part of the grid. Therefore, we did mesh control for these four transition points and set the width to height ratio of the square to 1.5, and the cell size to 0.2 mm, as shown in Figure 7.

### 2.3. Analysis

In the static stress analysis option, the solver type was set to iterative and large displacement was selected. At the same time, we used soft springs to stabilize the model or use inertial removal and set the contact mode to no penetration, so that the overlap of the pressure ring is prevented. Then, we run the static stress analysis; the operation process is shown in Figure 8.

The Mises stress, displacement, and deformation in the calculation results are shown in Figures 9–11. Among them, the iterative curve converges, indicating that the result was valid.

### 2.4. Clinical Curative Effects of the Designed Butterfly-Shaped Patellar Claw

#### 2.4.1. General Demographics of the Patients

A total of 27 cases were collected, including 17 males and 10 females, aged 16-57, with an average age of 39 years. The inclusion criteria were to select closed fresh patella fractures. Patients with mental illness and severe medical illness were excluded from this study. All cases were fresh fractures, including 21 cases of comminuted fractures and 6 cases of transverse fractures. According to Pengjian et al.'s fracture classification [12], there were 6 cases of type II, 6 cases of type IIIa, 13 cases of type IIIb, and 2 cases of type IIIc. All cases completed internal fixation within 3-10 days after injury. Written informed consent was obtained from all the patients included in this study.

#### 2.4.2. Clinical Procedures

After the patients were anesthetized (spinal anesthesia or combined spinal-epidural anesthesia), they were kept in the supine position, routinely sterilized the drape, and took the anterior patella longitudinal or transverse arc incision to reveal the patella fracture. Next, the joint cavity and fracture ends were cleaned up, the fracture was reset, and the ruptured anterior patellar ligament was sutured. The length of the patella was measured, and an appropriate model of a butterfly-shaped patellar claw was selected. The claw was put in sterile ice saltwater at 0~5°C and soaked for 2~3 minutes. Then, the compression ring was opened using the spreading forceps, and the upper and lower paw branches were opened using the needle holder, and a small incision was made in the corresponding quadriceps tendon and patellar ligament. According to the up-and-down method, first, the upper claw branch was hooked followed by the lower claw branch, and the position of the claw branch was adjusted to the right position. When the patellar claw was fit better on the surface of the patella and the patellar claw was fixed, the patella claw was poured with sterile hot saline (42°C), and the compression ring and claw branches of the patella claw were contracted and grasped the patella. Finally, after flexion and extension of the knee joint, it was assured that the fracture was firmly fixed, the joint movement was good, the incision was routinely closed, and the operation was completed.

#### 2.4.3. Postoperative Treatment

Postoperative compression and bandaging of the knee joint without external fixation. After anesthesia, the affected knee can be moved. On the second day after surgery, the patients were encouraged to get out of bed with crutches. The stitches were removed two weeks after the operation, and X-rays were taken regularly.

#### 2.4.4. Typical Case

This patient was a 16-year-old male. The main complaint was the swelling and pain of the left knee joint caused by a car accident, and the movement was restricted for 2 hours. X-ray film showed that the left patella was comminuted, fractured, separated, and displaced. On admission, the patient was diagnosed with a comminuted fracture of the left patella. The fracture classification was type IIIb. On the third day after admission, the operation of “left patella fracture open reduction and butterfly-shaped patellar internal fixation” was performed under combined spinal-epidural anesthesia. The fracture of the patella was revealed during the operation, and it was seen that the patella was a comminuted fracture, and there were many comminuted bones. After removing the blood clot at the fracture and the blood in the joint cavity, the fracture was reset, and the fracture was reset with a purse-string suture. A suitable model of butterfly patellar claw was chosen and soaked in sterile ice salt water for 2 to 3 minutes. The patellar claw was put on the patella according to the above-mentioned usage method and poured into the patellar claw with sterile hot saline (about 42°C). The compression ring of the patellar claw and the claw branch was contracted to grasp the patella. For the bone pieces that could not be “grabbed” by the lateral patellar claws, Kirschner wires were used to assist the fixation. After the intraoperative fixation was completed, the knee joint can was moved. The fracture was reduced, the patellar claw was firmly fixed, and the knee joint was able to be passively flexed and extended completely. On the second day after the operation, the patient was encouraged to move the knee joint and get out of bed with crutches and was discharged from the hospital after a week. The wound healed at the first stage, and the suture was removed two weeks after the operation.

#### 2.4.5. Analysis of the Curative Effect

The curative effect was evaluated according to Lu and Laitang's evaluation standard [13]. The patients were followed up to 15.5 months, and an average healing time was noted. Moreover, fracture displacement, loosening, fracture of internal fixation, or top abrasion caused by internal fixation was evaluated in all patients. The average time for all patients to get out of bed with crutches after surgery was noted. The curative effect was graded into the following categories:

*(1) Excellent: characterized by normal knee joint function, no pain, no muscle atrophy, free walking, no difficulty in stretching, and squatting*.

*(2) Good: knee joint function close to normal, no pain, mild muscle atrophy, walking freely, and squatting slightly worse*.

*(3) Acceptable: sometimes pain, muscle atrophy, and limited flexion, but greater than 90°, walking on flat ground without limp, and inconvenience in going up and down stairs and squatting.*

*(4) Poor: pain, muscle atrophy, less than 90° flexion, and inconvenience in squatting*.

#### 2.4.6. Reexamination and X-Rays

After internal fixation of the left patella fracture, the alignment was good, and the fracture line was blurred. One year later, the fracture was completely healed and the patient's left knee joint function was fully recovered. The patient requested to remove the internal fixation. When taken out, it was observed that the patellar claw was still firmly fixed on the patella, a thin layer of the dense membrane can be seen on the surface of the patellar claw, the tissue in the film that was attached to the patellar claw was smooth, and the surface of the patellar paw was also smooth. After taking it out, it was observed that there was no metal rust-like phenomenon such as blackening on the surface of the patella.

## 3. Results

### 3.1. Analysis of Mises Stress and Strain

The magnitude of the stress changes with the color of the graph is shown in Figure 9. The stress changes from small to large, and the color changes from blue-green to red. The red area is the maximum stress area (inside the compression ring); the maximum stress observed was 568.1 MPa (Figure 9). The *R* angle on the inner edge of the compression ring (marked in Figure 12) was a part that potentially could break, and its maximum strain was about 3.71*E* − 3. The red area was the most stressed part of the patellar claw. According to the performance indicators of TiNi memory alloy, the fully annealed fracture strength is 895 MPa (Table 2) [14]. It is worth noting that this is far greater than the 568.1 MPa stress experienced by the butterfly-shaped patellar claw. The maximum yield strength of the memory alloy material in the parent phase was 690 MPa, and the maximum stress value of the patellar claw was also less than this maximum value, so it was expected to show elastic deformation resistance within this range. Therefore, the butterfly-shaped patella claw was fixed on the patella, and it will not break when subjected to a force of 150 N on the encircling arm, and at the same time, there will be no pressure failure due to plastic deformation.

### 3.2. Deformation Displacement Analysis

The magnitude of the displacement changes with the color of the graph (as shown in Figure 10), the displacement changes from small to large, and the color changes from blue-green to red. The overall deformation of the patellar claw was 0.39 mm, and this deformation displacement was within the recovery range of the shape memory alloy. The mechanical performance and deformation of the patella claw under two different patella femoral joint forces (*F*_Q1_ and *F*_Q2_) at the angles of 30°, 60°, and 90° of knee flexion were analyzed. The respective *F*_Q_ were 367.5 N and 3675.0 N as shown in Table 1. Maximum displacements of deformation varied at different flexion angles suggesting that patella claw was preferable, with stronger resistance to tension and more stable antishearing force for clinical application.

### 3.3. Clinical Curative Effect

Reexamination of the X-rays when the patients were discharged from the hospital showed that the fractures were well aligned, the butterfly-shaped patellar claws were well positioned, and the fixation was firm. All patients' incisions healed by first intention. Of all 27 cases, 1 case lost follow-up after 9 months of follow-up, and the other 26 cases were followed up all the way. The average fracture healing time was 8-12 weeks, and the average follow-up time was 15.5 months. All patients had no fracture displacement, loosening, or fracture of internal fixation, and no top abrasion caused by internal fixation. All patients can get out of bed with crutches in 2~3 days after surgery, go to crutches in 2~4 weeks after surgery, go up and downstairs in 6~8 weeks, and take out the patellar claw in 11~13 months. Among them, there were 15 cases with excellent functional ratings, 10 cases with good ratings, 2 cases with acceptable ratings, and no cases with poor ratings.

## 4. Discussion

Patella fractures account for about 1% to 2% of all bone injuries [15]. Preserving the patella and restoring its normal anatomy and physiology as much as possible, giving strong internal fixation, early movement, and preventing the occurrence of traumatic arthritis are the basic principles for the treatment of various types of patella fractures [16].

In addition to stable shape memory effects, TiNi shape memory alloys also have the characteristics of superelasticity, low magnetic properties, fatigue resistance, wear resistance, corrosion resistance, and good biocompatibility. It is considered to be an excellent new bioengineering material and has been widely used in the medical field [17]. TiNi shape memory alloy patella claws have been used for many years in the treatment of patella fractures [18]. It conforms to the principle of tension band fixation, and the fixation is firm, and the effect is better for various types of patella fractures, especially comminuted fractures. In addition, it satisfies patients to perform early functional exercises after the operation, with fast functional recovery, and there is no phenomenon of K-wire rubbing after the operation. However, in clinical applications, we found the following: (1) intraoperative model selection is required to be accurate. In clinical applications, the selection is prone to be too large, resulting in insufficient compression between the ends or the selection is too small, which can easily cause the patella claw to fall off. (2) After the patella claw is fixed, sometimes the fracture line of the dorsal patella is wider. (3) During the intraoperative test, sometimes the two ends of the fracture may be slightly separated. Studies have reported that the selection of unsuitable patella concentrators or repeated heating and cooling causes loose fixation, slippage of the patellar claw, disengagement, local uplift, and deformity, and even redisplacement of fractures [17].

We believe that this is because the traditional fixation of the patellar claw is mainly based on the grasping and pressing of the two ends of the patella, while the pressure on the surface tension side of the patella is insufficient. After the knee joint is active, the surface tension stress is relatively large, and the top pressure of the two ends of the patella alone is not enough to offset the surface tension; thus, the fracture opens on the surface or the fracture line is wider.

The butterfly-shaped patella claw designs the waist of the traditional patella claw as a hollow dumbbell-shaped compression ring. In addition, we also use the characteristics of TiNi shape memory alloy to increase the overall longitudinal pressure while the patellar claw grasps the grip of the upper and lower paws. Therefore, the longitudinal compression effect between the fracture ends can be achieved to simulate the tension band effect of the patella surface ligament. The compression ring in the middle of the butterfly-shaped patella claw has the functions of [19]: (1) connect the upper and lower claws, which is equivalent to the waist of the traditional patella claws; (2) two wings are formed on both sides, covering the patella together with the upper and lower paw branches, increasing the enveloping area of the patella without affecting the blood supply, which is more advantageous for comminuted fractures; (3) tightly wrap on the patella through deformation to provide continuous fixed pressure; (4) the hollow design can reduce the stress shielding effect, facilitate the formation of callus, and shorten the healing cycle; (5) the hollow design facilitates the postoperative X-ray observation of fracture healing and prevents the radiopacity of the alloy material from blocking and observing it. The design of the claw branch is different from the curved design of the traditional patellar claw. The upper and lower branches of the butterfly-shaped patellar claw are straight, which is designed according to the physiological anatomical curvature of the patella, and the claws point to the center.

In the mechanical finite element analysis, we can see that the maximum stress that the compression ring of the butterfly-shaped patellar claw can withstand is 568.1 MPa. In this range, it always has elastic deformation resistance. The butterfly-shaped patella claw was fixed on the patella and will not break when subjected to a maximum force of 150 N on the encircling arm, and at the same time, there will be no pressure failure due to plastic deformation. Therefore, while completely offsetting the tension of the patella, it produces the unique memory resilience of the memory alloy and can convert the tension into pressure to produce a tension band effect, which provides effective stable fixation for early postoperative functional exercises. In actual clinical application, the model selection does not have to be very accurate. It has three models, which can meet clinical needs. We can choose a size of 2 smaller than the traditional shape memory alloy patella claw model. The installation method is basically the same as the traditional patellar claw. First, open the compression ring on the waist, and then open the upper and lower claws. Secondly, insert the upper claw branch, and then hook the lower claw branch into the lower pole of the patella. After correct installation, you can see that the butterfly-shaped patellar claw and the surface of the patella are more comfortable. After heating with warm salt water, contraction of the pressure ring can be seen. The obvious compression effect between the fracture ends can be observed from the hollow compression rings. After the fixation is completed, we can see that the fracture fixation is firmer when testing the knee joint movement. In addition, the intraoperative tests did not observe the slight separation of the two ends of the fracture and the opening of the dorsal side of the fracture. In particular, it has a better effect on comminuted fractures, especially stratified comminuted fractures. Before installing the patellar claw, the fracture should be reduced first, and the fractured piece should be fixed with a purse-string suture, and then the butterfly-shaped patellar claw should be fixed. For the crushed bone pieces that cannot be fixed by the claws, Kirschner wires can be used for auxiliary fixation. What is interesting is that it is easier to take out. It can be taken out after pouring a cold compress with ice saltwater. When we took it out, we noticed that the butterfly-shaped patellar claws were still firmly grasped without any signs of loosening. Its surface is wrapped by a layer of film, and the tissue in the film that is attached to the patellar claw is smooth, and the surface of the patellar claw is also smooth. After removal, there is no metal rust-like tissue on the surface of the patella, which may be due to the excellent wear resistance, corrosion resistance, and biocompatibility of the memory alloy.

Butterfly-shaped patellar claws are also inadequate. Our design is based on the traditional five-claw patellar claw design. However, if there are many crushed bones and the edge bones on both sides of the patella cannot be grasped and fixed, Kirschner wires, sutures, etc. are needed for auxiliary fixation.

## 5. Conclusion

The designed butterfly-shaped patella claws can provide an effective method for the treatment of patella fractures. The deformation and displacement analysis of the patella claw was in accordance with the biomechanical results needed in the clinic, and its stability can satisfy clinical requirements for early recovery. This study had some limitations including the following: the memory resilience of butterfly patellar claws under real working conditions could not be measured. Therefore, whether the restoring force of the compression ring and the claw branches can cause compression injury to the patella remains to be studied. Although there is an *R* angle on the inner edge of the pressure ring in the mechanical test, it is a part where fracture may occur. However, the maximum stress that NiTi memory alloy can withstand is much higher than the force of the human patella acting on the embracing arm. In addition, due to the small number of used cases, no cases of rupture have occurred yet, and further observation is needed by expanding the number of cases.

## Figures and Tables

**Figure 1:** The butterfly-shaped patellar claw.

**Figure 2:** Optimization model.

**Figure 3:** Material settings.

**Figure 4:** Constraint degree of freedom.

**Figure 5:** Set initial normal force.

**Figure 6:** Initial meshing.

**Figure 7:** Local mesh control.

**Figure 8:** Solution process.

**Figure 9:** Mises stress results.

**Figure 10:** Deformation displacement map.

**Figure 11:** Strain result.

**Figure 12:** Maximum force value of Mises stress.

**Table 1:** The force parameters of the patella at different knee flexion angles.

Force parameter	Knee bend angle (°)		
	30	60	90
Quadriceps tension *F*_1_/*N*	120.36	116.16	135.09
Patellar ligament tension *F*_2_/*N*	129.77	93.19	54.03
Patella joint force *F*_*q*/_*N*	*F*_Q1_ = 0.5, *G* = 367.5, *F*_Q2_ = 5, *G* = 3675.0		
Patellofemoral joint contact surface area *S* (mm^2^)	450.50	596.26	701.06
The ratio of patella joint force to body weight *K*	0.086	0.145	0.204

**Table 2:** Commonly used mechanical properties of nickel-titanium alloys.

Performance	Test results
Elastic modulus	Mother phase: 83GPa Martensite: 28-41 GPa
Poisson's ratio	0.33
Yield strength	Mother phase: 195-690 MPa Martensite: 70-140 MPa
Breaking strength	Fully annealed state: 895 MPa Work hardened state: 1900 MPa
Elongation at break	Fully annealed state: 25%-50% Work hardened state: 5%-10%
Stress concentration factor *K*_*t*_	8.5
Shape memory recovery rate	98%
Maximum recoverable strain	7.3%
Resilience	436.5 MPa
Fatigue life	1.4 × 10^7^ times
Nonlinear hyperelasticity	8.1%
Linear hyperelastic strain phase	4.3%
Damping performance (tan*δ*)	0.03 (completely austenite) 0.10 (complete martensite)

## Data Availability

The data used to support and prove the findings of this study are available from the corresponding author upon request.
